The article "Influence of Open Apex on Working Length Determination Using Cone-Beam Computed Tomography and Apex Locators: A Comparative In Vitro Study" was published in 2022. Journal: Biomed Res Int.

# Influence of Open Apex on Working Length Determination Using Cone-Beam Computed Tomography and Apex Locators: A Comparative In Vitro Study

**DOI:** 10.1155/2022/3811983

**Published:** 2022-07-23

**Authors:** Swati Srivastava, Hanan M. Alharbi, Mai Soliman, Elzahraa Eldwakhly, Manal M. Abdelhafeez

**Affiliations:** ^1^Department of Conservative Dental Sciences, College of Dentistry, Qassim University, Saudi Arabia; ^2^College of Dentistry, Qassim University, Saudi Arabia; ^3^Department of Clinical Dental Sciences, College of Dentistry, Princess Nourah bint Abdulrahman University, P.O. Box 84428, Riyadh 11671, Saudi Arabia; ^4^Faculty of Dentistry, October University for Modern Sciences and Arts, Egypt

## Abstract

**Objectives:**

The aim of this study is to assess the effect of open apex on working length (WL) determination with aid of cone-beam computed tomography (CBCT) and electronic apex locators (EALs).

**Methods:**

Thirty-two extracted human mandibular premolars were selected, and apical 5 mm was removed. Root canals were prepared from the apical to the coronal direction of the canal using peeso reamers up to size 5 (retrograde) to simulate open apex. The samples were analyzed by CBCT, and WL was established (CWL) by a radiologist. An endodontist prepared the access cavities, and visual working length (VWL) was recorded. The samples were embedded in a freshly mixed alginate mould up to cementoenamel junction. Each root canal length was measured with two different EALs—Root ZX mini and i Root. The measurements were repeated 3 times by using a digital caliper, and the mean was recorded by the endodontist who was blinded to the results of the CWL. The recorded data was statistically analyzed using the SPSS software.

**Results:**

The results of this study showed statistically significant difference between VWL and i Root, CWL and i Root, and Root ZX mini and i Root (*p* < 0.05). Amongst EALs, a superior accuracy was noted for Root ZX mini than as compared to i Root. However, no statistically significant difference was seen between Root ZX mini and CWL (*p* > 0.05).

**Conclusion:**

The present study showed that CWL is as accurate and reliable as VWL which is the gold standard. Amongst EALs, Root ZX mini performed more accurately than i Root. Preexisting CBCT scans should be used as an advantage in determining WL.

## 1. Introduction

Endodontic treatment has high success rate when it is done in correct manner including thorough debridement and perfectly done obturation [1]. The endodontic management of permanent teeth with immature apices poses a clinical challenge for oral health care practitioners. An open apex is an exceptionally wide apical foramen where achieving apical stop is challenging to be accomplished. The most favourable landmark to terminate the WL is the apical constriction. However, it lost in cases of immature apex. Steiner et al. [2] suggested that instrumentation of the apical portion of these canals must be avoided to prevent thinning of their fragile dentinal walls. There is therefore a requirement for clinical guidelines for WL determination in such teeth [3].

Predictable assessment of WL has been possible with the invention of EAL. The Root ZX has become the benchmark to which other EALs are compared. This instrument evaluates the quotient of the impedances of 2 frequencies (0.4 and 8 kHz) in order to identify the position of the file inside the canal. The Root ZX mini (J Morita, Tokyo, Japan) is a compact version of this device that exhibits similar functionality and accuracy [4].

i Root (S-Denti Co. Ltd, Seoul, Korea) apex locator has different frequencies—5 kHz and 500 Hz. The manufacturer claims that its accuracy is good, irrespective of canal contents. Despite having an accuracy of 80–90% in most root canals [2], their performance can be limited by multiple factors like the type of electrolytes in the canals and absence of apical constriction.

Various studies have noted that EALs give unreliable results in teeth with open apices [5, 6].

Inferable from their constraints, the use of EALs and radiographs ought to be enhanced with different strategies, particularly while treating extremely wide apical terminations. CBCT is validated as a tool for exploring root canal morphology in 3 dimensions, and in some studies, it was also used for estimating the WL. CBCT measurements in combination with EALs may also be useful for determining the WL [7].

To our knowledge, no previous study assessed the WL determination in an open apex using CBCT and EAL in an ex vivo model and compared it with gold standard of VWL. Therefore, the aim of the present study was to evaluate and compare the accuracy of WL determination in immature apices by using CBCT imaging and EAL against the gold standard. The null hypothesis was that there is no difference in the accuracy of WL determination using CBCT and EALs in an immature apex.

## 2. Methods

### 2.1. Sample Selection and Simulation of Open Apex

This study was approved by the Dental Research Ethics Committee (EA/F-4017-19) of the institution where it was conducted. Sample calculation was performed using 95% confidence interval to have a precision of 5%. Thirty-two extracted human mandibular premolars were selected. The inclusion criteria were single canal, completely formed apex, and absence of any preexisting restoration, caries, or morphologic defect. The exclusion criteria were teeth with any carious lesion, root resorption, fractures, immature apex, and calcification. Similar teeth with a length of 20 ± 0.51 mm were selected for standardization purpose. The samples were then immersed in 0.1% thymol solution for disinfection. The apical 5 mm of each tooth was removed using a low-speed diamond saw (SP1600, Wetzlar, Germany). These teeth were prepared from the apical to the coronal direction of the canal using peeso reamers up to size 5 (retrograde) to simulate immature teeth without any access cavity preparation.

### 2.2. Imaging Method and Evaluation of WL on the CBCT Scans

The teeth were numbered from one to thirty-two and randomly divided to be scanned by CBCT by placing four teeth at a time in premolar sockets of an artificial mandible. The mandible was covered with modelling wax. The CBCT unit used in this study was GALILEOS Comfort (Dentsply-Germany). It had a tube voltage of 85 kVp, tube current of 5-7 mA, field of view 15 × 15 × 15 cm^3^, isotropic voxel size 0.3-0.15 mm, and exposure time of 14 seconds to 2-6 seconds. Images were examined by using the scanner's proprietary software (Sidexis XG 3D Viewer; Germany) in an Intel Core i5-4460 at 3.20 GHz (Intel Corp, Santa Clara, CA) PC workstation running Windows XP professional SP-2 (Microsoft Corp, Redmond, WA). The sample teeth were adjusted in mesiodistal and buccolingual directions to obtain whole length in a single scan. WL was established by tracing a line in the centre from the occlusal reference point to the open apex. An average of mesiodistal WL and buccolingual WL was noted for each tooth as CWL. The examiner performing the CBCT measurements was a specialist in oral and maxillofacial radiology who exhibited routine experience in CBCT analyses for diagnostic purposes and was trained and calibrated by means of 10 samples before this investigation.

### 2.3. Access Opening and Visual WL Determination

Access cavities were prepared using endo access bur size 2 (Dentsply Maillefer, Ballaigues, Switzerland). The root canals were irrigated with 5 ml of 5% sodium hypochlorite. Next, barbed broaches were used to extirpate the remaining pulp. To avoid any canal enlargement, no root canal instruments were used. The actual length of the root canal was measured by inserting a size 15 K file in the canal until the file tip became visible at the open apex under 5x magnification using a dental operating microscope (S 100/OPMI pico; Carl Zeiss, Goeschwitzer, Germany). The silicone stop was placed at the reference point, and then, the file was removed from the canal. The distance from the base of the silicone stop to the file tip was measured with an electronic digital calliper. The measurements were recorded as the VWL which was taken as the gold standard in this study.

### 2.4. Embedding Samples in Alginate and EAL Measurements

The samples were embedded in a freshly mixed alginate mould up to cementoenamel junction. The labial clip was inserted into the mould simultaneously. Size 15 K file was clipped to the EAL, and electronic measurements were recorded with Root ZX mini (J Morita, Tokyo, Japan) and i Root (Meta systems Co., Seoul, Korea) according to the manufacturer's instructions in presence of saline. The EALs were used according to the manufacturer's instructions. For Root ZX mini, the file with a rubber stopper was advanced into the canal until an “APEX” reading was obtained; it was then withdrawn until the last green bar was reached. For i Root, the file was advanced until the EAL display indicated the “00” mark. All endodontic procedures were conducted by an experienced endodontist (8 years) who was blinded to the results of the CWL during the whole endodontic treatment.

### 2.5. Statistical Analysis

After data collection, data entry was performed in Excel. Data analysis was performed with the help of Statistical Package for Social Sciences version 22 (SPSS Inc, Chicago, IL). Nonparametric test was applied. Mann–Whitney *U* test was used to analyze the data with level of significance set at *p* < 0.05.

## 3. Results

The descriptive statistics of the mean values recorded in all the groups with the standard deviation (SD) is shown in Table 1. The intergroup comparison showed that the mean differences between VWL and CWL were statistically insignificant (*p* > 0.05). The mean differences between VWL and Root ZX mini were also found to be statistically insignificant (*p* > 0.05). The results of this study showed that i Root exhibited maximum significant difference when compared with the VWL, CWL, and Root ZX mini (*p* < 0.05) (Table 2). Amongst EAL, a superior accuracy was noted for Root ZX mini than as compared to i Root. However, no statistically significant difference was seen between Root ZX mini and CWL (*p* > 0.05).

The calculation of accuracy was done as percentage of recordings measured in each group which were within ±0.5 mm range of VWL. In the present study, we found an accuracy of 100% by CWL, 90% by Root ZX mini, and 70% by i Root within ±0.5 mm range of VWL (Figure 1). The CWL measurements are shown in Figure 2.

## 4. Discussion

The prognosis of any endodontic treatment depends upon the accuracy of the WL. Epidemiological studies show evidence on the good control over the WL as a prerequisite for a successful endodontic outcome [8, 9]. Histologic evidence has established optimal healing when there is minimal contact of root filling material and the periapical tissues [10]. During the developmental stage, an open apex can remain as a sequel to pulp necrosis following trauma or caries. It can also be created iatrogenically due to overinstrumentation or root resection. It remains as an exceptionally wide foramen where achieving apical stop remains difficult.

In the present study, single straight canals of mandibular premolars were assessed. The apex was instrumented with peeso reamers to obtain divergent open apex and mimic open apex as described by Gordon and Chandler [2]. The VWL was taken as the gold standard in this study.

The invention of EAL has led to a more predictable assessment of WL than as compared to conventional radiographs. Root ZX is one of the most extensively researched EALs and is the gold standard against which latest EALs are compared. Studies have shown that its accuracy varies from 50% to 100% [11–13]. Root ZX mini works on the same principle as Root ZX. In this study, Root ZX mini was found to be more precise EAL than i Root with an accuracy of 90%. It is a modification of third generation EALs. It works on the principle of comparative impedance or frequency. The difference in impedance from high (8 kHz) and low frequencies (400 Hz) at various sites in root canal helps Root ZX mini to establish the WL. This difference is least in coronal third, and it increases as the file goes to the apical third. Using the ratio technique, Root ZX mini presents an accurate indication of location of file [14].

For standardization purpose, the same K file size 15 was used for all the measurements. EALs are frequently used with small size files. However, the effect of file size in wider diameter canals is controversial in literature. A snug-fitting file is recommended to measure WL especially in the presence of blood [15]. In the present study, the apical 5 mm of the root was removed and then further enlarged from the apical to the coronal direction by peeso reamers up to size 5 (retrograde) to simulate immature apex. The mean differences between VWL and Root ZX mini were found to be statistically insignificant (*p* > 0.05) in this study. Our results are in corroboration with several studies which have reported accurate WL determination with the use of small size files in an open apex [15–17].

El Ayouti et al. [16] found that Root ZX was accurate, and the length measurements obtained with small and large size files were comparable in simulated open apex. However, they found that this accuracy with small K file sizes like #15 is not achieved in the presence of blood which may affect some of the variables in electronic root length determination. They found it to be accurate in presence of sodium hypochlorite. This could be one of the reasons for accurate results in our study with K file #15 in open apex with Root ZX mini which works with the same functionality and accuracy as Root ZX. Being highly electroconductive, sodium hypochlorite infiltrates into dentinal tubules [18, 19] and allows better electrical contact with the tissues.

The results of this study showed that i Root exhibited maximum significant difference when compared with the VWL, CWL, and Root ZX mini (*p* < 0.05) (Table 2). Amongst EALs, a superior accuracy was noted for Root ZX mini than as compared to i Root. This finding is in accordance with the literature where superior efficacy of Root ZX has been documented repeatedly.

The embedding media used in this study was alginate to simulate clinical conditions while evaluating the accuracy of EAL. Various other materials have been used in other studies like agar, gelatin, saline, and flower sponge. However, the performance of alginate was found to be superior for simulating periodontium. This can be attributed to its good electroconductive properties. It firmly supports the teeth and is economical and easy to handle [20]. It leads to an unbiased measurement as well. In this study, all the measurements were performed within 30 minutes as described by Topuz et al. [21] to prevent dehydration of alginate.

Despite having 80-90% accuracy of EAL in WL measurement, their performance is limited by many factors like absence or presence of apical constriction [2]. CBCT scanning has become prominent in endodontics for diagnosis and treatment planning. They provide clinicians with WL measurements that are comparable with the gold standard VWL. Studies have shown that it is a consistent and reliable tool for measuring WL with high precision [22, 23]. Moreover, it has advantage of less radiation and possible 3-D evaluation. The results of this study demonstrate that CBCT scans can be used alternatively for estimating the WL in teeth with open apex. It has been reported in literature that EAL can give unpredictable results in various conditions like presence of metallic restorations which lead to electrical short circuiting, size of apical foramen, type and size of measuring file, irrigation solution used, and electroconductivity of the pulp [24]. In such cases, clinician can take advantage of any preexisting CBCT scans of patients which can aid in estimating precise WL. This can improve the endodontic prognosis of teeth with immature apex.

The findings from the present study should not be used as an indication of CBCT scanning for estimating the WL in immature apex. Adhering to ALARA (as low as reasonably achievable) principle [25, 26], only cases having preexisting CBCT scans taken for diagnosis can be used. The null hypothesis was acceptable for CWL and Root ZX mini. However, it was rejected for measurements taken with i Root. Attempt to simulate open apex in a clinical scenario was tried to make as precise as possible; however, there may be some variations.

The present study showed that CWL is as accurate and reliable as VWL which is the gold standard. However, in reality, the availability of CBCT units in all dental set-ups throughout the world might be challenging. Moreover, the patients with open apex might not be having any preexisting CBCT records. According to the findings of the present study, we recommend the use of Root ZX mini EAL in open apex cases to get accurate results when preexisting CBCT scans are not available due to any of the aforementioned reasons.

The limitation of the current study was the absence of blood due an in vitro set-up. This might not be true in a clinical scenario where blood and possibly pus or serum can be present which might give inaccurate readings on Root ZX mini in cases of open apex. Future studies can target a larger sample size in vivo and determine the outcomes of this study.

## 5. Conclusion

Amongst EALs, Root ZX mini performed more accurately than i Root. Preexisting CBCT scans are of advantage to the clinician in determining the WL in cases of open apex.

## Figures and Tables

**Figure 1:** Accuracy of CWL, Root ZX mini, and i Root when compared with VWL as shown in the bar diagram.

**Figure 2:** WL measurement of mandibular premolars using CBCT imaging (CWL).

**Table 1:** Descriptive statistics of the mean values of WL including minimum and maximum values recorded in different groups.

Groups	*n*	Mean + SD (*n* = 32)	Minimum	Maximum
VWL	32	16.05 ± 0.83^A^	13.20	18.72
CWL	32	16.02 + 0.94^A^	13.25	18.80
Root ZX mini	32	16.03 ± 0.79A	13.16	18.64
i Root	32	14.3 ± 1.25^B^	11.21	19.23

**Table 2:** Mean difference between VWL and WL recorded by different EAL.

Groups	*n*	Mean difference (SD)
CWL	32	0.0^A^
Root ZX mini	32	0.25 (0.26)^A^
i Root	32	1.90 (0.31)^B^

Different superscript uppercase letters in the same column indicate a statistically significant difference (*p* < 0.05). The same superscript indicates insignificant difference (*p* > 0.05).

## Data Availability

The data presented in this study are available on request from the corresponding author.
